RETRACTED

# Wireless sensor network-based machine learning framework for smart cities in intelligent waste management

**DOI:** 10.1016/j.heliyon.2024.e36271

**Published:** 2024-08-15

**Authors:** Karan Belsare, Manwinder Singh, Anudeep Gandam, Varakumari Samudrala, Rajesh Singh, Naglaa F. Soliman, Sudipta Das, Abeer D. Algarni

**Affiliations:** a School of Electronics and Electrical Engineering, Lovely Professional University, Phagwara, Punjab, 144411, India; b School of Computer Science and Engineering, Lovely Professional University, Phagwara, Punjab, 144411, India; c Department of Electronics and Communication Engineering, NRI Institute of Technology, Agiripalli, Vijayawada, Andhra Pradesh, 521212, India; d Division of Research and Innovation, Uttaranchal University, Dehradun, Uttrakhand, 248007, India; e Department of Information Technology, College of Computer and Information Sciences, Princess Nourah bint Abdulrahman University, P.O. Box 84428, Riyadh, 11671, Saudi Arabia; f Department of Electronics and Communication Engineering, IMPS College of Engineering and Technology, Malda, 732103, West Bengal, India

**Keywords:** Internet of things, Machine learning, Smart waste management system, Wireless sensor network

## Abstract

Environmental safety is one of the key issues that are directly related to a country's prosperity**.** One of the most fundamental aspects of a sustainable economy is waste management and recycling. Better recycling safety and efficiency may be achieved via the use of intelligent devices rather than manual effort. In this research, we describe a machine learning-based architecture for smart trash collection and sorting using the Internet of Things and wireless sensor networks. The goal of this study was to develop an autonomous method for producing an efficient and intelligent waste parameter monitoring system for a novel waste management system, using the Internet of Things (IoT) and Long Range (LoRa) technologies. Several possibilities are explored, all of which may be applied to the development of the three nodes. The number of trash cans, garbage stench, air quality, weight, smoke levels, and waste categories are all tracked in real-time via the Internet of Things and the Thing Speak Cloud Platform, which can be set up in numerous places. In the end, a fog layer-deployed intelligent waste classification framework consists mostly of four layers: input, feature, classification, and output. Using the Thrash Box dataset, the proposed system develops a categorization method into trash classes such as household, medical, and electronic garbage, in addition to object identification. Traditional machine learning methods, such as the multi-kernel support vector machine (SVM) and the Adaboost ensemble classifier, are employed in the classification layer, while the Resnet-101 deep convolutional neural network model is used in the feature layer. Experiments were conducted to evaluate the suggested method's ability to classify garbage and provide accurate predictions about their respective categories. Compared to other state-of-the-art models, the suggested method's performance was shown to be superior in the presented trials.

RETRACTED

## 1 Introduction

Waste categorization is an integral aspect of the first step in responsible waste management. Greater consumption is a direct result of a growing population [1]. It also causes an increase in waste. Garbage may be produced in two main settings: the household and the workplace. Correctly sorting garbage has positive effects on both the environment and the economy. Trash that is properly sorted helps conserve resources and protect the ecosystem as a whole [2]. The necessity for further training on categorization makes it challenging to apply regulations. As a result, teaching people about the dangers of trash and the correct way to get rid of it is essential. Studies have shown that throwing out a lot of trash from the kitchen, including a lot of plastic bags, may have a terrible effect on the environment. Uncollected garbage can pollute water supplies and soil, cause the release of toxic gases, and reduce agricultural yields, among other negative effects. The conventional methods of waste sorting have many drawbacks, including the need for human intervention, limited efficiency, and poor quality. The use of deep learning (DL) methods for trash classification is gaining traction in the academic community [3].

The most effective method of combating pollution is to implement a waste management system based on machine learning (ML) and the Internet of Things (IoT). These technologies provide accurate data on trash and the best path for garbage trucks, accelerating the pace at which rubbish is collected and decreasing the total time it takes to collect garbage [[4], [5], [6], [7], [8]]. Poor scheduling is to blame for the current waste management systems' failure to meet expectations since garbage collectors often forget that they are supposed to pick up the trash. Furthermore, they have no idea where the drop-off will occur. One prominent use is the fact that IoT innovation has become a potent instrument for fostering thriving urban communities. Rapid urban population expansion has led to an increase in waste production, which is a serious challenge for every modern city. The combination of ML and IoT represents a promising direction for waste management research. The number of interconnected gadgets in IoT is expanding rapidly to provide the required waste management features. As a result, there is a rise in the volume of data being collected, which in turn motivates the adoption of ML techniques to boost the responsiveness and functionality of software [9,10]. In most uses of Wireless Sensor Networks (WSNs), knowing where things are is essential. There have been several recent presentations of localization algorithms, however, most of them only deal with problems in a single dimension. However, this is a challenging issue in three-dimensional applications because of the wide range of heights present. The sensors are set in the mountains to monitor traffic in certain areas and the air to monitor pollution levels. In these contexts, 2D localization models are not accurate. Consequently, creating 3D localization algorithms for WSNs presents significant challenges [11,12].

RETRACTED

The ability of computers to pick up new skills and make independent judgements is a key feature of artificial intelligence (AI), and this is where ML comes in. In academia, researchers in the discipline of machine learning investigate various statistical approaches and models. Since it offers the most cutting-edge capabilities in the realm of computing, ML has reached its apex of popularity. This also applies to other forms of machine learning, such as deep learning [[13], [14], [15], [16]]. CNNs, or convolutional neural networks, are a key component of deep learning. CNN has shown amazing progress in the field of image recognition. They are typically employed in tandem with picture classification to evaluate visual content. They are essential for a wide variety of applications, from Facebook's photo tagging to driverless cars. They're putting in long hours behind the scenes, helping with everything from healthcare to security. In this study, we provide a garbage-based picture classification and tagging system [[17], [18], [19], [20], [21], [22], [23], [24]] that draws on these ideas. The garbage image classification hybrid learning module made it possible to train and evaluate the created models after the appropriate data sets had been prepared.

The contributions of this article are summarized as follows.

• Developed Data Acquisition and Monitoring Framework Using Wireless Sensor Networks and Thing Speak IoT Analytics for Waste Management
• Designed the hybrid learning garbage waste classification system architecture.
• Feature layer from pre-trained ResNet 101 and classification layer from machine learning algorithms are implemented to train and test garbage waste images.
• A visual garbage classification system integrating image classification and object detection.

RETRACTED

This article is arranged into five sections. Section 2 describes the overview of related contributions; section 3 presents the overall material and methods used in the implementation process. Section 4 depicts the experimental results of our proposed system along with related discussion. Finally, section 5 illustrates the conclusion of this manuscript.

## 2 Related work

RecycleNet employs a carefully calibrated deep CNN architecture to categorize certain sorts of recyclable items. In this research, we present a framework for a waste management system [25] that incorporates AI and IoT. The smart waste management system [26] was developed by using a deep learning model and LoRa communication protocol. In this study, we explore the use of a deep learning convolutional neural network for trash categorization, which combines methods from image classification and object recognition [27]. The CNN algorithm [28] facilitates waste classification. Trash sorting into useful categories like "organic" and "recyclable" has been made easier with the use of deep learning algorithms [29]. We provide a deep-learning automatic trash classification method [30] to enhance the efficiency of initial garbage pickup. To address the issue of litter in public areas, we present a multilayer hybrid DL system (MHS) [31] to automatically classify rubbish. An approach to waste identification that can be used on mobile devices and help solve rubbish problems in cities [32]. In Ref. [[33], [34]], we provide a method for developing intelligent systems that make use of DNN and other forms of machine learning. In place of the conventional waste management system [35], smart segregation makes use of IoT devices, DL algorithms, and Image Processing technology. For application in futuristic metropolises [36], we develop a novel intelligent DRL-based model for recycling waste item detection and classification (IDRL-RWODC).

Using CNNs and an uneven precision measurement weighting strategy (UPMWS), we introduce a novel ensemble learning model called EnCNN-UPMWS [37] for the classification of HSW using waste pictures. In Ref. [38], we observe a trash sorting system built using a combination of the TensorFlow object detection model, the SSD MobileNet V2 model and the Arduino microcontroller. A system is demonstrated that can automatically separate recyclables, food waste, and hazardous materials without the intervention of a person. Deep learning algorithms are utilized to identify and categorize garbage; recyclable and organic wastes are then sorted for future utilisation [5]. An intelligent garbage sorting system is developed using the ResNet-50 CNN model [6]. According to Ref. [7], a multi-model cascaded CNN (MCCNN) is recommended for trash picture recognition and classification. Using IoT devices, an automated waste sorting system was created [8]. DDR-net (Double fused Deep CNN using ResNext) [10] is an enhanced version of the ResNext model that takes advantage of double fusion and regularization. A trash sorting system that uses transfer learning and a basic neural network [11]. The suggested hardware solution is a deep-learning-based implementation of image categorization using a CNN System Architecture in a Real-time embedded system. When it comes to garbage, SmartBin can separate biodegradable items from the rest [12]. For the suggested deep learning-based classification approach to medical waste identification and categorization [13], the ResNeXt deep neural network is provided as a practical example of a DNN. The goal of this research is to create a garbage-type-identifying image classifier based on a CNN [14]. In this study, we suggest a hybrid approach to garbage classification that might be implemented in a smart trash classification model that operates in real-time [15]. Garbage sorting using a neural network and image processing [16]. The garbage classification Deep Learning Networks are trained using a dataset that combines user-generated data with garbage Net [39,40]. The Smart Waste Management and Categorization Method, State-of-the-Art Categorization Approach. A deep learning-powered unmanned aerial vehicle (UAV) garbage-scanning system [[17], [18], [19], [20]]. They proposed automating the garbage classification issue with ML and DL techniques in Refs. [[18], [19], [20], [21], [22], [23], [24]].

RETRACTED

## 3 Material and methods

The proposed model is focused on a typical IoT layered architecture for waste management. The generalized framework has mainly a four-layer architecture which is composed of application, middleware, network, and perception layers which are discussed and shown in Fig. 1, and the working flow is given in Fig. 2.

**Fig. 1:** Generalized IoT framework for waste monitoring.

**Fig. 2:** Proposed architectural scenario.

Each layer has its significance and plays an important role in justifying the working of the proposed model. In the perception layer, nodes are deployed which sense the data from sensors and transfer it to the network layer. In the network layer, data received from the perception layer is transferred to the middleware layer using Wi-Fi and LoRa technology based on IoT. In the middleware layer, data analytics is applied to received data from the perception layer which provides intelligent control at the perception layer and respective data decisions at the application layer. In the application layer, data received from the perception layer is monitored in real-time at cloud services to show the real-time activity and status of nodes. Further, these layers are discussed below.

RETRACTED

### 3.1 Perception layer

This layer, which relies heavily on hardware, collects data from the physical world, processes it, and then transmits the results across encrypted channels to higher levels of the system. Physical characteristics, toxic gas levels, rubbish levels, garbage images captured by the camera, etc. are all detected using specialized sensors, and item identification data is collected as a byproduct.

A wireless sensor network–based scenario, as depicted in Fig. 2, is proposed as part of the smart city's design considering the IoT-based framework in trash monitoring for intelligent waste management.

Here, it is assumed that there are three societies in which the first two nodes are deployed in societies where it senses the parameter from the dustbin to which sensors are attached, and the third node is deployed in a dumping station where all waste materials are collected, sorted using data analytics model by taking pictures from the camera and processed further for decomposition as per their waste category. The first node is set up with an infrared (IR) sensor, an odour (Odour) sensor, and an air quality (Air Quality) sensor, all of which are interfaced with the microcontroller on the node's board. The second society makes use of a Node 2 equipped with a Weight sensor and a Smoke sensor, all of which are interfaced with the Node MCU microcontroller. The ESP 32 Node MCU is used as the main microcontroller in both nodes, a series of low-cost, low-power systems on a chip microcontroller with integrated Wi-Fi and dual-mode Bluetooth. With the NodeMCU-ESP32, comfortable prototyping is possible by configuring with simple programming via the Arduino IDE. Finally, in the third civilization, the camera is set up at the third node, a dumping station where a circulating conveyor belt mechanism is installed. Once the trash is placed on it, a camera installed on it captures the image and sends it to the middleware layer for data analysis using an analytics model. The analytics model predicts the type of waste category and provides a control signal to the dumping station to sort materials as per the type of thrash which is discussed in the next section. Several sensor components are used in both nodes, Node1 and Node2 as shown above in Fig. 2, mainly IR Sensor, Odour Sensor, Air Quality Sensor, Weight Sensor, and Smoke Sensor are discussed below.

#### 3.1.1 Proximity IR E18 sensor

An infrared proximity sensor called E18 IR is employed to detect the presence of industrial objects. It is a cheap, simple-to-assemble sensor that barely interferes with the ambient lights and environment. It is a non-contact, variable range-detecting sensor. It includes a transmitter and receiver in a single-module configuration. A modulated IR signal is emitted by the transmitter and reflected by anything in its sight or path. The transmitter receives the reflected signal, which then outputs a digital signal to the microcontroller. A digital output is produced by the non-contact detecting sensor whenever an object enters a predetermined range. The sensing range of the sensor is 3–80 cm. In real time accuracy of detecting distance varies from ± 1 to 2 cm.

RETRACTED

#### 3.1.2 Odour sensor

Carbon monoxide (CO) odour sensors are designed to detect specific odours. MQ7 is used for odour sensors. The sensor measures CO levels in the air. This sensor offers quick response time and great sensitivity. Analog resistance is the sensor's output. The sensitivity of the sensor is ≥ 3 %.

#### 3.1.3 Air Quality Sensor

Sensors that measure air quality find airborne impurities, including substances that could be unsafe to living beings, such as particles, contaminants, and toxic gases. The MQ 135 air sensor monitors air quality and can detect CO2, aiding in maintaining a safe atmosphere on the premises. The sensor has a fast response and recovery time with adjustable sensitivity as per the threshold defined for the application.

#### 3.1.4 Weight sensor

A weight sensor determines the garbage bin's weight. A particular kind of transducer is a weight transducer, often known as a weight sensor. It transforms a mechanical force applied as an input, such as weight, load, tension, pressure, or compression, into another physical variable. The calibrated rated output of the sensor is 1.0 ± 0.1 mV/V.

#### 3.1.5 Smoke sensor

An instrument that detects smoke, usually as a fire indicator, is called a smoke sensor. Industries can use the Gas Sensor MQ2 to find gas leaks. The detection range of this gadget includes H2, CH4, LPG, CO, smoke, alcohol, and propane. This sensor has good sensitivity to combustible gas in a wide range of ppm.

### 3.2 Network layer

This layer, which makes use of Infrared, GSM, ZigBee, Wi-Fi, and LoRa, oversees sending the measured data from the perception to the middleware layer, where the expert services are installed. The network layer also handles data management and cloud computing tasks in addition to its basic responsibilities. In the IoT system, communications protocols are also included and enable easy data sharing. Low-power devices that use TCP/IP for seamless data exchange are represented by the messaging protocol standards known as Message Queue Telemetry Transport (MQTT).

RETRACTED

To help enhance the nodes' battery life and network capacity, LoRa also includes an adaptive data rate mechanism. The LoRa protocol has several numbers of layers, including device, application levels, and encryption enabling secure communications in the network. Specifically, radio bands designated for industrial, scientific, and medical (ISM) uses are used by the low-power LoRa protocol, which is designed to function over long distances using unlicensed spectrum. Although the accessible bands are limited and certain countries have severe regulations regarding how frequently a device on these bands may transmit, LoRa devices communicate at sub-gigahertz frequencies, enabling long-range data transfer. IoT messaging is standardized through the MQTT protocol. A scalable and dependable method of connecting devices via the Internet is the MQTT publish/subscribe protocol, which is standardized by OASIS and ISO. It is a simple protocol made for publishing and receiving messages. It uses less power and has very little bandwidth requirement.

### 3.3 Middleware layer

This software layer or maybe a group of sublayers acts as an interpreter to facilitate communication between otherwise incompatible IoT components. Communication between the application layer and the perception layer is essential, and this is made possible through concurrency. Machine learning is the primary method of data analysis in this context. The fog layer is another name for this layer. Thanks to the IoT fog layers, systems may now perform necessary processing and analysis as close to the data's original location as feasible. We have built an analytics model for a trash categorization system in this tier. Based on the data acquisition from three nodes data, primarily analytics model is divided based on the camera sensor from node 3 and sensor data from node 1 and node 2. Two analytics models are developed, first, Camera Sensor Data Analytics for Classification of Waste Images, and second, Sensor Data Analytics Using Supervised Machine Learning Modelling.

#### 3.3.1 Camera Sensor Data Analytics for Classification of Waste Images

The waste object of garbage is the focus of the processing, analysis, and classification phases of the garbage waste classification system. The training and testing phases make up the entirety of the recognition system method. Fig. 3 is a simple representation of a categorization system that has been presented. The suggested system begins with the same pre-processing and feature extraction processes at the beginning of both the training and testing phases.

**Fig. 3:** Framework for waste classification.

RETRACTED

##### 3.3.1.1 Trash Box dataset

Trash Box [19] stocked with junk from different settings. Domestic, medical, and electronic garbage were the primary categories used to categorize the photographs in the Trash Box. Future, Table 1 describes how these classes are broken down into subclasses to make it easier to differentiate between different types of garbage items and to promote future study in this area. To make a Trash Box, we first gathered photographs of common waste items by doing a thorough online search.

**Table 1:** Thrash box dataset – class-wise statistics.

Thrash Class	Sub-classes	No of Images	Total
Domestic Waste	News Papers	200	4476
	Paper Tissues	1062	
	Paper Cups	639	
	Bottles	571	
	Bags	504	
	Spray Cans	500	
	Beverage Cans	1000	
Medical Waste	Syringes	507	2010
	Surgical Gloves	496	
	Surgical Masks	500	
	Medicines	507	
E-Waste	Electronic chips	615	3437
	Laptops and Smartphones	774	
	Appliances	926	
	Electric wires	568	
	cords and cables	554	

##### 3.3.1.2 Pre-trained Resnet-101 deep convolutional neural network model

To assess images, the proposed method employs a deep convolutional neural network (resnet-101). In feature extraction, the representational power of a deep network is put to one of its simplest and most immediately useful uses. To start, we input a network that has already been trained to recognize several different object categories from many images. Therefore, the model has been educated to represent several image types, each with its own unique set of attributes. The network generates a tree diagram to represent the images it is given. Features at a higher level are layered on top of features at a lower level. To acquire the feature representations of the images, activations on the network's last layer, the global pooling layer, are required. The output features are a unified representation of the input characteristics across all geographic areas in the layer. ResNet-101 is a deep-learning network consisting of 101 convolutional layers. Residual neural networks (ResNets) are an example of an ANN that is inspired by the architecture of pyramidal cells in the brain. Residual neural networks accomplish this by using skip connections, or shortcuts, to skip over certain layers. Nonlinearities (ReLU) and batch normalization are common components of ResNet models, which are often constructed with double or triple-layer skips in between. HighwayNets are a type of model that needs an additional weight matrix to learn to skip weights. In modelling, "Dense Nets" refer to models with numerous parallel skips. A neural network that does not generate residuals is known as a non-residual network or simple network. ResNet was inspired by VGG-19, another basic network architecture with 34 layers, to which we also provided a direct link. ResNet, short for "residual network," is an essential tool for addressing issues in computer vision. ResNet101's [14] convolutional layers consist of 33-layer blocks, and 29 of those squares are recycled into later layers. The ImageNet dataset, which includes 1000 different classes of objects, was used to first train this network. The structural plan of the pioneering design is shown in Fig. 4. This graphic shows how the input images are partitioned into residual blocks, with each block consisting of many layers. This may be expressed mathematically as.

RETRACTED

**Fig. 4:** ResNet 101 deep learning model [20].

Consider,

Source Domain, DS = {(γ1S, ρ1S), …., (γiS,ρiS), …‥, (γnS, ρnS)} with learning task LS, LD, (γmS, ρmS) ∈ R;

Target Domain, DT = {(γ1T, ρ1T), …., (γiT,ρiT), …‥, (γnT,ρnT)} with learning task LT, (γnT,ρnT) ∈ R;

(m, n) is the training data sizes where n ≪ m and ρ1D and ρ1T are the labels of training data. Then the TL is represented as shown in below Equation (1):

(1) DS = DT, LD = LT

##### 3.3.1.3 Machine learning-based classification model

To provide expected output in the form of a waste type and additional object type of trash, the classification of garbage waste using two machine learning classifiers was carried out throughout the train, validate, and test stages. In this study, we make use of the robust and adaptable machine learning classifier techniques. To get the best results from classification hyperparameter tweaking, K-fold validation (K = 10) is used. Because the model's performance depends on the values of the hyperparameters, this is crucial information. Once the trained model has been validated, it will be able to make predictions about the output label of the dataset.

When applied to feature space instead of input space, a kernelized SVM is functionally like a linear SVM. The idea is to first do a nonlinear mapping of the data into feature space before applying a linear SVM. The kernel technique is utilized in a kernelized SVM, therefore the real procedure looks different. The kernel function (K), which returns the dot product of two representations of features, defines the mapping between the data and feature space implicitly. Let's pretend that x and x′ are input space points. Then, we can write down the ‘K’ as shown in Equation (2) below,

(2) K(x,x′) = Φ(x)⋅Φ(x′)

Where Φ is a function that maps the input space to the feature space.

**Table:** 

Algorithm 1: Implementation of SVM Algorithm
Step 1: Initialize the input feature vector and output target vector.
Step 2: Select the appropriate kernel function.
Step 3: Defining the parameters and constraints.
Step 4: Solve the optimization problem to find the optimal hyperplane.
Step 5: Make predictions based on the learned model.

RETRACTED

One type of ensemble boosting classifier, Ada-boost, or Adaptive Boosting, is an iterative ensemble approach. The AdaBoost classifier combines numerous weak classifiers to create one robust classifier with high accuracy. The goal of Adaboost is to train a data sample and adjust the classifiers' weights in such a way that out-of-the-ordinary data is reliably predicted. The following can be used to assign initial weights (W) as depicted in Equation (3):

(3) W = 1/ N ∈ [0.1]

N represents the total number of observations. meaning the total number of files. The real impact might be categorized by α as shown in Equation (4).

(4) α = 0.5 ln ((1-TotalError)/Total Error)

Where alpha represents how much weight a certain stump has in the whole process. The number of incorrectly labeled records is the overall inaccuracy. The following formula can be used to revise the sample weights as formulated in Equation (5).

(5) W_i_ = W_i-1_*e^+-^ α

In this case, the updated sample weight is calculated by multiplying the original sample weight by Euler's number. If the data are correctly categorized, alpha will be positive; otherwise, it will be negative.

**Table:** 

Algorithm 2: Implementation of AdaBoost Algorithm
Step 1: To begin, each data point is treated equally.
Step 2: A model analysis is built and performed on a sample of data.
Step 3: This model is used to make inferences over the whole dataset.
Step 4: Errors are computed by comparing predicted values to observed ones.
Step 5: Data points that were inaccurately predicted are given more weight when building the model.
Step 6: The error value can then be used to assign weights. For instance, an observation may be given greater credence if it has a larger margin of error.
Step 7: Once the error function has stabilized, or the maximum number of estimators has been achieved, the procedure begins again.

#### 3.3.2 Sensor Data Analytics Using Supervised Machine Learning Modelling

The proposed sensor data analytics to generate the control signal for controlling the actuators of the hardware system using supervised machine learning is depicted in Fig. 5. The proposed framework begins with data feature engineering, feature dataset splitting, and machine learning modeling for result prediction.

**Fig. 5:** Garbage waste classification framework.

##### 3.3.2.1 Acquired sensed data

A prototype hardware-based system is used to implement the proposed experimental architecture, and this system has undergone extensive testing. The acquired dataset has the feature attribute of waste detection level using IR sensor (cm), Odour level (ppm), Air quality level (ppm), weight of smart dustbin (gm) and Smoke Level (ppm) for two different nodes. For node1, the actuator control for dustbin is represented by dustbin status and poisonous waste status. For node2, the actuator control for dustbin is represented by dustbin status and harmful gas status. This dataset includes hourly readings recorded over the course of many days and under a variety of weather situations.

RETRACTED

##### 3.3.2.2 Data feature engineering

Data transformation into machine-learning-friendly features is called "feature engineering." To improve the quality and performance of ML models, feature selection, extraction, and transformation are performed. The quality of the characteristics used to train ML models is crucial to the success of those models. These methods improve the machine learning model's ability to learn from data by drawing attention to the most relevant patterns and correlations in the data.

One definition of a feature variable in the context of machine learning is a discrete, quantifiable quality or characteristic of a data item that serves as input to a machine learning algorithm. Features are data representations that can be either numeric, categorical or even textual, depending on the nature of the problem at hand. In most machine learning algorithms, cleaning and transforming data are prerequisite processes. The process of "data cleansing" entails finding and fixing any mistakes or inconsistencies in the data collection. This process is crucial for ensuring the data is correct and trustworthy. The purpose of data transformation is to make the variables in a dataset more amenable to machine learning by transforming and scaling them. Methods like log transformation, standardization, and normalization may be used.

##### 3.3.2.3 Feature dataset splitting

In feature splitting, one variable is divided into several smaller ones. This is commonly done when a variable comprises sub-components that can be better analyzed independently. The term "feature split" refers to the process of dividing a feature into sub-features. A dating feature, for instance, may be broken down further into its parts (year, month, and day). Machine learning models can benefit from this since more data details are captured. The dataset is split into two parts: the training set and the testing set. The standard split is 70 % for training and 30 % for testing, however, this might change based on the size of the dataset and the specific application.

##### 3.3.2.4 Machine learning modelling

To provide expected output in the form of a waste type and additional object type of trash, the classification of garbage waste using two machine learning classifiers was carried out throughout the train, validate, and test stages. In this proposed study, we make use of the robust and adaptable machine learning classifier techniques in which two machine learning algorithms are used, Decision Tree Bagging (DTB) and K-Nearest Neighbor (KNN) supervise machine learning algorithms. To get the best results from classification hyperparameter tweaking, K-fold validation (K = 10) is used. This is very important since the model's output is sensitive to the values of the hyperparameters. Predictions regarding the dataset's output label can be made by the trained model once it has been verified.

RETRACTED

The benefits of the suggested algorithms are further forth below. When the gap between classes is manageable, KNN does similarly well. It works well in settings with several dimensions. When the number of dimensions exceeds the number of samples, this method excels. DTB is a classifier that is simple to implement since it requires less hyperparameter tuning than competing techniques. DTB improves the performance of inefficient ML models. DTB is resistant to overfitting since it sequentially executes models with related weights.

##### 3.3.2.5 Algorithm steps

**Table:** 

Algorithm 3: Data Analytics Considering Sensor's Data
***Input:****Two nodes sensor data, odour (in ppm), air quality (in ppm), smart dustbin weight (in gramme), and smoke levels (in ppm)*
***Output:****Control signal for actuators*
***Procedure:***
*Step1:* Prepare the sensor's dataset containing various attributes of the sensor data
*Step2:* Split the sensor dataset into train and test into 70-30 % ration
*Step3:* Apply data pre-processing operation on both the train and test set
*Step4:* Select the pre-processed features from the train and test set
*Step5:* Prepare the train and test set features dataset for training of model and result prediction
*Step6:* Initialize the input feature vector and output target vector for training
*Step7:* Selecting the appropriate hyperparameters for both machine learning classification model
*Step8:* Train and validate the model using finetuning of the classifier
*Step9:* Load the trained model for each classifier
*Step 10:* Make predictions based on the learned model to get the prediction for the control signal for actuators.

### 3.4 Application layer

While the application layer may not always contribute directly to the development of the IoT architecture, it is at this level that numerous services are developed that link with consumers, making this the level at which the data is interpreted and made available. This level is responsible for the development of graphs and business models. Waste data in real time may be tracked and analyzed with the aid of this additional layer.

RETRACTED

## 4 Experimental results and discussion

### 4.1 Data acquisition and monitoring framework

The proposed architectural framework makes use of elements typical of IoT layer-wise design. Node 1 and node 2 employ sensors connected to the open-source Node MCU platform to track environmental data at closed and open waste facilities, respectively. The shield and microcontroller that the smart devices use to communicate with one another are linked. The Arduino Integrated Development Environment (IDE) may be utilized to build embedded C applications for acquiring sensor data. This information is sent wirelessly via the LoRa protocol and IEEE 802.11 Wi-Fi. The coordinator may access the cloud server from anywhere with Wi-Fi access. The perception layer, seen in Fig. 6, collects data from sensors, analyses it, and stores it in a database until it can be sent to the Thing Talk Cloud platform through the MQTT protocol. Fig. 7 depicts the experimental setup as it is planned. As can be seen in Fig. 8, the Thing-Speak cloud platform makes use of a graphical user interface (GUI) dashboard to present information on a mobile device or monitoring screen.

**Fig. 6:** Data handshaking with Thing Speak Cloud Platform.

**Fig. 7:** Experimental setup.

**Fig. 8:** Thing Speak Dashboard with other sensing Data Representation.

To assess the system's performance in multiple ecological tasks, wearable sensor parameters are tracked, researched, and analyzed. When examining normal and abnormal circumstances in the same domain, the sensor reading parameters are monitored for two different sensor nodes placed in an open and closed environment.

The distributions are represented statistically on the cloud. An alert is issued to the appropriate supervisor or responsible person for each anomaly discovered in values that meet the given threshold.

The sensed data from two sensor nodes is monitored in real-time on a serial monitor with time stamp values as shown in Fig. 9.

**Fig. 9:** Sensor's output on serial monitors with timestamp values.

As discussed in section 3.1, all sensors’ data is sensed and acquired using Node MCU ESP 32 microcontrollers, over a period of 100 days. The mean value plot of distance using IR sensor, odour level, air quality level, weight level and smoke level data parameter for each day is shown in Fig. 10, Fig. 11, Fig. 12, Fig. 13, Fig. 14, in which periodic data is collected at the different conditional waste environments.

**Fig. 10:** IR sensor data.

**Fig. 11:** Odour level data.

RETRACTED

**Fig. 12:** Air quality level data.

**Fig. 13:** Weight sensor data.

**Fig. 14:** Smoke Sensor data.

Fig. 10 represents the data that indicates the level of waste in cm, the threshold defined in blue colour categorizes the level of waste, above the threshold level acts as no waste is found in the dustbin.

Fig. 11 depicts that data shown in black colour is represented as safe and red is represented as unsafe for various discrete events under environmental conditions for the odour Sensor and the threshold mentioned in blue colour acts as the threshold which discretizes the safe and unsafe values.

Fig. 12 depicts that data shown in black color is represented as safe and red is represented as unsafe for various discrete events under environmental conditions for Air Quality Sensor and the threshold mentioned in blue colour acts as a threshold that discretizes the safe and unsafe values.

The weight sensor data is represented in Fig. 13. The value of weight above the threshold acts as the weight of the dustbin in grams of various waste collected and below the threshold indicates the minimal weight.

Fig. 14 depicts that data shown in black color is represented as safe and red is represented as unsafe for various discrete events under environmental conditions for Smoke Sensor and the threshold mentioned in blue colour acts as the threshold which discretized the safe and unsafe values.

The mean values of different waste condition parameters are shown in Table 2, Table 3 for abnormal and normal activities over a day using sensor monitoring anomaly detection, which lowers the cost of maintenance for smart waste management.

**Table 2:** Sensor Parameters Mean values at node 1 for day hours.

Sensors Parameter	Unit of Measurement	Threshold Value	Mean Value	
			Abnormal	Normal
IR sensor	*Cm*	50	32.53	80.8
Odour Sensor	Ppm	250	363.79	121.73
Air Quality Sensor	Ppm	200	319.27	119.43

**Table 3:** Sensor Parameters Mean values at node 2 for day hours.

Sensors Parameter	Unit of Measurement	Threshold Value	Mean Value	
			Abnormal	Normal
Weight Sensor	Gm	1000	2256.66	374.42
Smoke Sensor	Ppm	230	357.69	109.9

As compared to existing work developed by various authors, formulated in Table 4, based on the sensor used for development and technology used to build the system, our proposed model is much superior in all aspects.

**Table 4:** Comparative analysis table.

Parameters		References				
		Gunawan T. et al. [3]	T. Bakhshi et al. [32]	Dev V. Savla et al. [5]	Shamin.N et al. [34]	Proposed Model
**Sensors Used**	Ultrasonic/IR	✓	✓	✓	✓	✓
	Odour			✓		✓
	Air Quality			✓	✓	✓
	Weight	✓				✓
	Smoke			✓		✓
**Technology Used**	IoT	✓	✓	✓	✓	✓
	LoRa					✓
	Fog Intelligence		✓	✓	✓	✓
	Real-Time Statistics	✓	✓	✓	✓	✓
	Notification/Alert System					✓

RETRACTED

### 4.2 Camera Sensor Data Analytics for Classification of Waste Images

This section analyses the suggested categorization model. Domestic garbage, medical waste, and electronic waste make up the bulk of the typical benchmark dataset utilized in experimental settings. These studies were conducted using a Windows laptop equipped with a core i5 CPU and 8 GB of RAM running MATLAB R2018b. Several images from a common benchmark dataset have been extracted and organized into three semantic categories for this collection. Fig. 15, Fig. 16, Fig. 17 display some examples of the photographs we used.

**Fig. 15:** Images of Class I i.e., Domestic Waste.

**Fig. 16:** Images of Class II i.e., Medical Waste.

**Fig. 17:** Images of Class III i.e., E-waste.

All images are full colour and have been downsized to a 256x256 resolution. In the suggested model, a 70-30 % ratio is used for training and testing of the model. Multi-kernel SVM and Adaboost classifiers are employed as the two-classifier models in the proposed experiment. Hyper-parameter optimization based on a grid search is used to tune the hyperparameters of training. The confusion matrix is used to evaluate all performance metrics. The quality of the job has been evaluated using a confusion matrix and the performance assessment criteria. The effectiveness of an algorithm is typically displayed in the form of a table, called an error matrix or supervised learning error table. Table 5 shows the results of a performance evaluation of the two algorithms in terms of the amount of time needed to classify each of the three categories. Training and testing the classification step with Ada boosting algorithms took longer, as seen in Fig. 18.

**Table 5:** Performance evaluation time.

Classification Phases	Training Time (sec)		Testing Time (sec)	
	MK-SVM	AdaBoost	MK-SVM	AdaBoost
Category I	81.54	90.16	35.90	42.46
Category II	64.89	78.48	29.27	32.85
Category III	89.41	93.71	39.50	45.37

**Fig. 18:** Process evaluation time.

The classification performance parameters, sensitivity, specificity, and f-score are evaluated for three primary waste category classifications for both algorithms and mentioned in Table 6, Table 7, Table 8 respectively. Each category has various output labels or classes as per the type of waste categories described in Fig. 19, Fig. 20 for both algorithms for category I, domestic type of waste classification respectively. It is observed that some waste category classes are classified with maximum performance for both algorithms.

**Table 6:** Classification report performance for category I.

Output Classes	Classification Algorithms					
	MK-SVM			AdaBoost		
	Sensitivity	Specificity	F-score	Sensitivity	Specificity	F-score
News Papers	86.95	100	97.08	69.56	99.17	77.66
Paper Tissues	86.36	99.18	83.33	27.27	97.74	33.33
Paper Cups	89.28	99.58	91.91	46.42	95.02	36.93
Bottles	96.29	99.79	96.29	66.66	99.17	78.26
Bags	88.23	100	97.40	70.58	99.39	77.92
Spray Cans	77.27	99.59	86.73	45.45	98.77	58.13
Beverage Cans	85.71	100	96.77	71.42	99.39	75.75

RETRACTED

**Table 7:** Classification report performance for category II.

Output Classes	Classification Algorithms					
	MK-SVM			AdaBoost		
	Sensitivity	Specificity	F-score	Sensitivity	Specificity	F-score
Syringes	72.72	99.82	88.88	77.27	99.31	80.18
Surgical Gloves	45.71	97.18	49.07	54.28	95.07	42.60
Surgical Masks	63.15	93.80	43.79	52.63	93.62	38.16
Medicines	61.29	97.02	54.28	32.25	97.20	37.03

**Table 8:** Classification report performance for category III.

Output Classes	Classification Algorithms					
	MK-SVM			AdaBoost		
	Sensitivity	Specificity	F-score	Sensitivity	Specificity	F-score
Electronic chips	82.05	96.75	78.81	79.48	94.58	69.50
Laptops and Smartphones	80	98.28	80	92	96.56	73.24
Appliances	97.36	99.64	97.36	100	99.64	97.93
Electric wires	53.33	100	85.10	60	100	88.23
cords and cables	78.94	100	94.93	63.15	99.66	84.50

**Fig. 19:** Performance of Category I using MK-SVM.

**Fig. 20:** Performance of Category I using AdaBoost.

Similarly, for the classification of category II, various output labels or classes as per the type of waste categories are described in Fig. 21, Fig. 22 for both algorithms. It is observed that some waste image classes are classified with better performance of specificity rate for both algorithms. The classification of categories III with various output labels is shown in Fig. 23, Fig. 24 for both algorithms.

**Fig. 21:** Performance of Category II using MK-SVM.

**Fig. 22:** Performance of Category II using AdaBoost.

**Fig. 23:** Performance of Category III using MK-SVM.

**Fig. 24:** Performance of Category III using AdaBoost.

Table 6, Table 7, Table 8 show the classification performance of domestic, medical and e-waste classes. In each class, several thrash materials are predicted using an analytics model to show their prediction accuracy by using sensitivity, specificity, and f-score parameters. The intelligent models are trained for each category and their subclasses represent the thrash material component.

At the last, the result analysis performance of an algorithm is analyzed and compared with existing standard work shown in Table 9 and it is found that the proposed method is found to be efficient in terms of accuracy with 94.1 %.

**Table 9:** Comparative analysis of performance.

References	Accuracy (%)
Recycle Net [1]	81
EnCNN-UPMWS [25]	92.85
SVM [26]	87
Proposed Method	94.1

RETRACTED

### 4.3 Sensor Data Analytics Using Supervised Machine Learning Modelling

A prototype hardware-based system is used to implement the suggested experimental architecture, and this system has undergone extensive testing. Two nodes' odour (in ppm), air quality (in ppm), smart dustbin weight (in gramme), and smoke levels (in ppm) are among the feature attributes included in the collected data set. The dustbin status and the presence of toxic waste serve as the actuator control for the dustbin at node 1. The presence or absence of dust and toxic gases, respectively, serve as actuator controls for node 2's trash can. This dataset includes hourly readings recorded for many days and under a variety of weather situations. The average daily value for each sensor's characteristic. Building a sensor net for smart waste management with the use of supervised machine learning algorithms, and developing fundamental models embedded systems for successful waste management, are the two main stages of experimentation. The same hardware configuration is utilized as discussed earlier. The MATLAB Integrated Development Environment (IDE) and the MATLAB Statistics and Machine Learning Toolbox (SMT) were used to write the model's code. The effectiveness of the system is measured using a confusion matrix. The confusion matrix parameters are used to determine the accuracy, specificity, sensitivity, and f-score of the proposed model. The model was trained and tested with MATLAB's built-in statistics and machine learning tools, and two supervised machine learning models, KNN and Decision Tree Bagger (DTB) classifier. For optimal model training, both techniques necessitate the best possible hyper-parameters, which may be found through a grid search. Table 10, Table 11 show the results of running the classification model on both nodes of the system. Fig. 25, Fig. 26, Fig. 27, Fig. 28 depicts the results of a comparison of the accuracy, sensitivity, specificity, and f-score of two different classifiers applied to two different actuator controllers.

**Table 10:** Performance evaluation of classification model for Node 1 System.

Attributes	Accuracy (%)		Sensitivity (%)		Specificity (%)		F-score (%)	
	DTB	KNN	DTB	KNN	DTB	KNN	DTB	KNN
Actuator 1	86.66	76.66	81.81	77.27	100	75	95.74	86.73
Actuator 2	96.66	70	100	89.47	90.90	36.36	95.95	73.91

**Table 11:** Performance evaluation of classification model for Node 2 System.

Attributes	Accuracy (%)		Sensitivity (%)		Specificity (%)		F-score (%)	
	DTB	KNN	DTB	KNN	DTB	KNN	DTB	KNN
Actuator 1	84.50	72.85	79.81	74.80	98.5	76.15	92.90	84.45
Actuator 2	93.75	71.15	98.60	85.45	87.30	38.05	93.35	71.80

RETRACTED

**Fig. 25:** Accuracy performance statistics.

**Fig. 26:** Sensitivity performance statistics.

**Fig. 27:** Specificity performance statistics.

**Fig. 28:** F-score performance statistics.

## 5 Conclusions and future scope

• The issues of waste segregation and management are ever-present and have far-reaching consequences for the environment. Modern waste management may be streamlined with the right application of technology.
• The Internet of Things is a cutting-edge innovation that will make every city on Earth ultra-modern and efficient. The fast development of smart cities has also led to an increase in waste production. Waste management in the Internet of Things is a major issue.
• To collect information on raw thrash material in real-time via the Internet of Things, the proposed system made use of the ThingSpeak cloud platform. In addition, this study also recommended adopting LoRa for trash monitoring in places where an internet connection cannot reach. The given solution met all the requirements established during the testing of the proposed system.
• In addition, the proposed system is implemented at the middleware layer for the data analytics system, where data is collected periodically for dataset creation from sensors and cameras.
• The proposed intelligent model used hybrid learning approaches which are useful for addressing the problem of waste material classification.
• The proposed approach is the most accurate of the methods compared by a wide margin with an overall accuracy rate of 94.1 % for the camera-based analytics model and 90.39 % for the sensor-based data analytics model.
• Further, the use of deep learning algorithms with large data collection will have future implications. There is still a space for improvement in the efficiency of trash classification.
• By improving the data set, we may potentially make the future cleaner and more aesthetically pleasing, which would lessen the burden on the sanitation department and its employees and speed up the garbage sorting process.

## Funding

This research was funded by 10.13039/501100004242Princess Nourah bint Abdulrahman University Researchers Supporting Project number (PNURSP2024R51), Princess Nourah bint Abdulrahman University, Riyadh, Saudi Arabia.

## Data availability statement

The data presented in this research are available on request from the corresponding author.

## CRediT authorship contribution statement

**Karan Belsare:** Writing – original draft, Software, Investigation, Formal analysis, Conceptualization. **Manwinder Singh:** Writing – original draft, Supervision, Investigation, Data curation, Conceptualization. **Anudeep Gandam:** Writing – original draft, Validation, Supervision, Resources, Conceptualization. **Varakumari Samudrala:** Writing – review & editing, Visualization, Validation, Methodology, Investigation. **Rajesh Singh:** Writing – original draft, Software, Resources, Data curation, Conceptualization. **Naglaa F. Soliman:** Writing – review & editing, Project administration, Methodology, Funding acquisition, Formal analysis. **Sudipta Das:** Writing – review & editing, Visualization, Methodology, Formal analysis, Data curation. **Abeer D. Algarni:** Writing – review & editing, Software, Project administration, Funding acquisition.

RETRACTED

## Declaration of competing interest

The authors declare that they have no known competing financial interests or personal relationships that could have appeared to influence the work reported in this paper.
